This article has been retracted.

# The Influence of the Development of the Internet of Things Industry on the Optimization of the High- and New-Tech Industry Structure under the Wireless Mobile Network

**DOI:** 10.1155/2022/7257688

**Published:** 2022-07-18

**Authors:** Yu Liu, Zhengchao Zhang, Shicao Jiang, Yawen Yang

**Affiliations:** ^1^School of Economics and Management, Liaoning University of Technology, Jinzhou 121000, Liaoning, China; ^2^School of Economics, Bohai University, Jinzhou 121000, Liaoning, China; ^3^Sunwah International Business School, Liaoning University, Shenyang 110136, Liaoning, China

## Abstract

At present, the pressure on China's economic development is increasing day by day due to the profound changes in the internal and external environment. The global economic pattern is undergoing significant changes in terms of the external environment. Adjusting and optimizing the industrial structure will aid in achieving the goal of facilitating transformation through steady growth in the short term. Meanwhile, it will also accelerate sustainable economic development. In this study, the relevant theories of industrial structure optimization are described based on the impact of wireless mobile networks and the Internet of things (IoT) industry. Based on the gray correlation degree, the high- and new-tech industries under the development of the IoT industry are analyzed and the impact of optimization of the high- and new-tech industry structure is investigated. The results show that the development of the IoT industry has driven the development of the high- and new-tech industry. The gray correlation between the development of the IoT industry and the high- and new-tech industry obtained is 0.64, indicating a strong correlation. The average output share of the electronic computer and office equipment manufacturing industries is 47.09%. The average output ratio of the industrial structure optimization of the electronics and communication manufacturing industry is 42.55%. Moreover, the proportion of the output of medical manufacturing and medical equipment and instrument manufacturing industrial structure optimization is small, 15.63% and 10.54%, respectively. The results have significant value in the research on the impact of the development of the IoT industry on the high- and new-tech industry under the wireless mobile network and the effect of its industrial structure optimization.

## 1. Introduction

The new generation of communication technology is developing rapidly. The central issue is the development of the basic network, which is the foundation of the information society. Accelerating the construction of a broadband network is essential for economic transformation and sustainable economic development in the future [1]. The Internet of things (IoT) is a new paradigm that allows electrical devices and sensors to communicate with each other over the Internet to make our lives easier. The industrial structure-based IoT technology includes chip design, application equipment, system integration and software, telecom operators, and service providers. The terminals are countless devices or items. Therefore, a large market space can be derived from the IoT [2]. The IoT industry belongs to the tertiary industry and also the high- and new-tech industry. From the perspective of industrial structure optimization and upgrading, the structure of this industry is gradually optimized from low to high [3]. For example, in terms of enterprise operating costs, if radiofrequency identification (RFID) technology is used, the entire enterprise can be automated. Enterprises can reduce the error rate and automatically correct product information errors in all aspects of product production [4]. Moreover, detailed product information is recorded to improve the operational efficiency of enterprises. The global retail giant Walmart in the United States adopts RFID technology for all commodities, and Walmart saves 8.35 billion US dollars every year, most of which are labor costs. RFID technology can help solve two of the biggest challenges in retail: out of stock and wastage. Walmart can ensure that its logistics supply chain is smooth and unobstructed through RFID tag technology [5]. The characteristics of the IoT industry's development are consistent with the need for China's industrial structure to be optimized and upgraded. The IoT industry's rapid expansion has increased the proportion of IoT output value in total societal output value year after year. The Internet of things (IoT) will play a significant role in China's economic development [6].

International Business Machines Corporation (IBM) of the United States released the smarter earth strategy. It proposed to embed sensors in various objects and connect them to form the IoT [7]. The IoT was united through supercomputers, thereby realizing the integration of people and things. Its essence was to use a more intelligent method to change the way people communicate with each other. Information technology was used to increase flexibility and efficiency. The European Union (EU) carried out innovative work on IoT technologies and applications [8, 9]. The EU hoped to lead the development of the IoT in the world. At the Global IoT Conference in 2009, senior EU experts introduced the “EU IoT Action Plan” to various countries [10]. In the EU, operators and equipment manufacturers were active, in promoting the development of machine-to-machine (M2M) technology and services [11, 12]. Japan announced its national informatization strategy based on the IoT in 2004 [13]. The core of the Japanese strategy was people-oriented, realizing various information connections between people and things [14]. Japan adopted a more reasonable adjustment and combination of social resources to realize this strategy. Japan hoped to create a more developed digital network society and make Japan the standard for future world social development. In this way, it could ensure its favorable competitive position while solving social problems [15, 16]. Some foreign researchers proposed a model to study structural changes and economic growth. To benefit smart city applications, Khajenasiri et al. [17] conducted a survey on IoT systems for smart energy control. He remarked that IoT is currently being used in only a few application areas to benefit both technology and people. IoT has a very broad scope, and in the near future, it will be able to cover practically all application areas. Li et al. [18] developed a dynamic strategy for data-centric IoT applications. The need for a suitable device, software configuration, and infrastructure necessitates cost-effective solutions to support a large number of IoT applications running on cloud platforms. Developers and academics working on IoT solutions are taking into account both huge platforms and the heterogeneous architecture of IoT items and devices. The author in [19] stated that interoperability is important in the Internet of things since it allows the integration of devices and services from several heterogeneous platforms to deliver an efficient and dependable solution. Several more studies [20–22] focused on the importance of interoperability and explored the issues that interoperability in the IoT faces. Climate change was addressed by Kim et al. [23], who presented an IoT-based ecological monitoring system. Existing procedures, according to Tey, are time-consuming and require a lot of human engagement. A routine visit is also required to collect data from the sensors installed at the investigation site. The IoT can be used to explore the preservation of the propensity for endogenous economic growth in the industrialization of a country's economy [24]. In 2008, domestic scholars compared the basis of the three industrial structures in Jiangsu, Zhejiang, and Shanghai. They analyzed the precise positioning of the industrial structure adjustment in Zhejiang Province and proposed a rational industrial structure path that conforms to the industrial layout of Zhejiang Province [25].

IoT developers and researchers are working together to extend the technology on large scale and to assist society to the highest possible level. However, developments are possible only if we study the various limitations in the present technical methods. In this study, the influence of the development of the IoT industry on the optimization of the high- and new-tech industry structure is analyzed and the relevant theories of industrial structure optimization are described based on the impact of wireless mobile networks on the IoT industry. According to the gray correlation degree, the high- and new-tech industries under the development of the IoT industry are investigated and the impact of the optimization of the high- and new-tech industry structure is studied.

The rest of the manuscript is organized as follows: Section 2 provides an overview of the optimization of the structure of high-tech industries. In Section 3, different results are presented, and Section 4 concludes the manuscript.

## 2. Optimization of the Structure of High-Tech Industries

### 2.1. IoT Industry under Wireless Mobile Network

The fundamental way to change the mode of economic development in the new period is to remove development obstacles and accelerate the optimization of industrial structure. This is certainly fantastic news for IoT businesses and the industry as a whole. It will also encourage businesses to undergo industrial transformations. The next generation of communication technology is continually evolving, but the creation of the basic network remains a major challenge. This is the foundation of the information society. Accelerating broadband construction is essential for economic transformation and sustainable economic development in the future. The structure of the wireless mobile network is shown in Figure 1.

The wireless access network is responsible for connecting the terminal to the communication network and corresponds to the terminal and the base station part. Between the base stations and the Internet is the core network. It primarily serves as an operational support system for end-user mobility, session management, and service management. The bearer network is the foundational network that connects the wireless access network to the core network. It is mainly responsible for data transmission. It is located between the wireless access network and the core network. The wireless access network, bearer network, and core network work together to form the pipeline of mobile communication [26].  Figure 2 demonstrates wireless resource management.

The coverage, capacity, and quality of service (QoS) are the three pillars of wireless network performance. They influence and interact with each other. Radio resource management ensures the quality of service, maximizes coverage, and improves spectrum utilization efficiency. It seeks the best working balance between coverage, capacity, and quality [27]. Information sensing device consists of sensors, radiofrequency identification technology, global positioning systems, infrared sensors, laser scanners, and gas sensors. The IoT refers to the real-time collection of any object or process that needs to be monitored, connected, and interacted with through various information sensing devices. It also collects information on sound, light, heat, electricity, mechanics, chemistry, biology, and location, among other things. It will be simple to identify, manage, and govern the connections between things, things and people, and all things and the network.  Figure 3 shows the three layers of the IoT.

The three layers of the IoT are comprehensive perception, reliable delivery, and intelligent processing. The IoT is formed based on sensing devices and the Internet. Perception devices are equivalent to various sensors, while RFID is equivalent to passive sensors. The Internet is formed under the integration of the communication network, the Internet, and the broadcasting network, and the IoT is formed by the integration of various sensors and the three networks. The IoT is formed based on sensing devices and the Internet. Perception devices are equivalent to various sensors, while RFID is equivalent to passive sensors. The Internet is formed under the integration of the communication network, the Internet, and the broadcasting network, and the IoT is formed by the integration of various sensors and the three networks. The development of sensors will accelerate the development of a “Smart Planet.” The promotion of “Smarter Planet” will accelerate the development of sensors. Therefore, the “IoT” must be a booming emerging industry, making production and life intelligent driven by computers, communication systems, sensors, and software. The development of the information industry and the needs of human society prove that the IoT is the result of industrial development and an inevitable requirement for mankind to pursue a smart society [28].

### 2.2. The Mechanism of IoT to Promote the Optimization of Industrial Structure

The IoT industry is one of the foundations of the information industry. The development of the IoT industry and the application of IoT technology have effectively promoted the transformation of the industrial structure to the “three-two-one” pattern. The development of the IoT has become a positive driving force for the optimization and upgrading of the industrial structure. Therefore, the optimization of the industrial structure must be accelerated in response to the development of the IoT industry. The theoretical foundation of the development of the IoT industry is shown in Figure 4.

The theoretical basis of the development of the IoT industry includes the theory of technological innovation, industrial correlation, sustainable development, and industrial structure optimization. The main body of innovation in the theory of technological innovation is the “entrepreneur.” Entrepreneurs' innovative activities are the main reason for the rise and development of technological innovation. The premise of technological innovation is the development of the IoT. The understanding of the IoT continues to deepen across industries. The development concepts of “first networking, then adding value” and “building the IoT industry development ecology with the platform as the core” have gradually formed a consensus in the industry, which has led to the rapid deployment of the IoT networks and platforms [29]. The good expectations of the market have optimized the scale deployment of the IoT wide area network, and the network technology has continued to breakthrough. In the industrial relevance theory, the direct consumption degree of producing a certain product to another product is the direct energy consumption coefficient. The equation is computed as follows:

(1) $$\begin{array}{c} a_{i,j}=\frac{q_{i,j}}{Q_{j}},i,j=1,2,\;n, \end{array}$$

where *a*_*i*,*j*_ is the direct energy consumption coefficient. *q*_*i*,*j*_ is the product *i* as a direct intermediate input. *Q*_*j*_ is the total output of product *j.* (2) is the mathematical model of physical input-output without total labor output.

(2) $$\begin{array}{c} AQ+Y=Q, \end{array}$$

where *A* is the direct energy consumption coefficient matrix. *Q* is a column vector consisting of the total output of various products. *Y* is a column vector of final product compositions. The following equation is obtained by the matrix transformation of (2):

(3) $$\begin{array}{c} Q={\left(I-A\right)}^{-1}Y, \end{array}$$

where social production planning can be implemented by computing the (*I*-*A*) inverse matrix. The degree to which an industry affects other industries is the industry influence coefficient. Its equation is as follows:

(4) $$\begin{array}{c} q=\frac{a_{l}}{\bar{A_{w}}}, \end{array}$$

where *a*_*l*_ is the mean value of the column coefficient of the inverse matrix of the industry. $\bar{A_{l}}$ shows the average value of the column coefficients of the inverse matrix of all industries. *q* > 1 means that the industry's influence is above the average level in all industries. *q* = 1 indicates that the industry's influence is at an average level in all industries. *q* < 1 means that the industry's influence is below the average level in all industries. The degree to which an industry is affected by other industries is the industry sensitivity coefficient. It can be expressed as follows:

(5) $$\begin{array}{c} p=\frac{a_{w}}{\bar{A_{w}}}. \end{array}$$

In (5), *a*_*w*_ is the mean value of the horizontal coefficient of the inverse matrix of the industry. $\bar{A_{w}}$ is the average value of the mean value of the horizontal coefficient of the inverse matrix of all industries. The industry sensitivity coefficient *p* is consistent with the feedback of the industry influence coefficient. The generalized economic development cost function in sustainable development theory is shown as follows:

(6) $$\begin{array}{c} C=M+Cd+Cs, \end{array}$$

where *M* is the production cost. It is also an intermediate input, which is determined by the level of technology. *Cd* is the cost of economic development when dealing with the relationship between man and nature. *Cs* is the cost incurred in dealing with the relationship between people. The economic development cost in the narrow sense is studied from the definition of sustainable development. It refers to the economic development cost of the relationship between man and nature, ecological cost, environmental cost, and resource capital. The expression is shown as follows:

(7) $$\begin{array}{c} Cd=Cs+Ce+Cr, \end{array}$$

where *Cs* is the ecological cost. *Ce* is the environmental cost. *Cr* is the resource cost. Minimization of economic costs is to achieve the minimization of individual costs. It is the rationalization of the discount rate of ecological, environmental, and resource utilization. Industrial structure optimization refers to the process of promoting the rationalization and advanced development of the industrial structure. The process of industrial structure optimization includes adjusting the supply and demand structures that influence the transformation of the industrial structure via government-sanctioned industrial policies. Therefore, the optimal allocation and reallocation of resources are realized, and the rationalization and advanced development of the industrial structure are promoted. The optimization of industrial structure is a rationalization process in which the economic and technological connection and quantity proportional relationship between industries change from uncoordinated to coordinate. It is also a process in which the industrial structure evolves from a low level to a high level.  Figure 5 reveals the content of industrial structure optimization.

The supply structure refers to the supply ratio of capital, labor, technology, and natural resources as production factors in various industries of the national economy under certain price conditions. It is also the industrial relationship that is connected by this supply relationship, including capital structure, investment structure as a supply factor, labor supply structure, technology supply structure, resource endowment, natural conditions, and resource supply structure. Demand structure refers to the proportion of demand for products or services of various industries that the government, enterprises, households, or individuals can undertake under a certain income level. It is also the industrial associations linked by this demand. International trade structure refers to the proportion of imports and exports of products or services in various industries of the national economy and the industrial associations linked by this import and export relationship. International investment structure refers to the proportion of domestic investment and foreign investment. It is also the proportion of domestic investment in different industries and the proportion of foreign investment in different industries in the country and various derived structural indicators.  Table 1 shows the mechanism of industrial structure optimization.

### 2.3. The Role of the Development of the IoT Industry on the Optimization of the Structure of High- and New-Tech Industries

The predecessor of high and new technology is high technology. It arose in the 1940s with the use of nuclear energy and the advent of electronic computers. The high- and new-tech industry is the same as the high-tech industry. As a special term, it has more practical value than academic value. Therefore, it has many definitions. High- and new-tech industries and high-tech industries are interchangeable, and it usually refers to a technology-intensive bureau formed from upstream to downstream of a certain technology. Also, emerging industries with short life cycles are defined differently in Western countries [30]. High- and new-tech industry generally refers to emerging industry groups with high technology intensity, fast update speed, and high added value. It can effectively save resources and energy and play a leading role in related industries.  Figure 6 shows the role of the development of the IoT industry in optimizing the structure of the high- and new-tech industry.

The development of the IoT industry has promoted the development of the high- and new-tech industry economy. It also optimizes the structure of the high- and new-tech industry. The gray correlation degree is used to analyze the relationship between the development of the IoT under the wireless mobile network and the factors of the optimization of the high- and new-tech industry. The important factors that affect the target value are found, and the main characteristics of things are grasped. The following equation is the calculation method of the correlation coefficient.

(8) $$\begin{array}{c} \;\xi_{i}\left(k\right)=\frac{\underset{i}{\min}\left({△}_{i}\left(\min\right)\right)+0.5\underset{i}{\max}\left({△}_{i}\left(\max\right)\right)}{\left|x_{0}\left(k\right)-x_{i}\left(k\right)\right|+0.5\underset{i}{\max}\left({△}_{i}\left(\max\right)\right)}, \end{array}$$

where *ξ*_*i*_(*k*) represents the relative difference between the comparison curve *x*_*i*_ and the reference curve *x*_0_ at the *k*th time. 0.5 is the resolution factor. The following equation is the expression of the degree of association.

(9) $$\begin{array}{c} r_{i}=\frac{1}{N}\overset{N}{\underset{k=1}{\sum }}\xi_{i}\left(k\right), \end{array}$$

where *r*_*i*_ is the correlation degree between the IoT industry variable and the high- and new-tech industry structure variable. *N* is the number of data. The following equation displays the industry dependency representation:

(10) $$\begin{array}{c} d_{i}=\underset{l}{\sum }w_{l}\;d_{i}^{l}, \end{array}$$

where *d*_*i*_ is the dependency of the industry. *w*_*l*_ is the weight vector of the index. *d*_*i*_^*l*^ is the result of the normalization of the gray correlation degree by the industry.

## 3. Results and Discussion

### 3.1. Analysis of the Impact of the Added Value of the Total Output Value of the High-Tech Industry

High- and new-tech industry is divided into medical equipment and instrument manufacturing, electronic computer and office equipment manufacturing, electronics and communication manufacturing, aerospace equipment manufacturing, and medical manufacturing. The total output value structure of the high- and new-tech industry from 2016 to 2021 is revealed in Figure 7.

The electronics and communication manufacturing industry accounts for the highest proportion of the total output value of the high- and new-tech industries from 2016 to 2021, with an average value of 51.15%. The total output value of the electronic computer and office equipment manufacturing industry ranks second, with an average proportion of 27.86%. Similarly, the total output value of the medical manufacturing industry is 13.30%. Likewise, the total output value of medical equipment and instrument manufacturing reported is 5.33%. In addition, the aerospace equipment manufacturing industry accounts for the lowest proportion at 2.42%. The results indicate that the total output value of the aerospace equipment manufacturing industry is the lowest in the technology industry of colleges and universities.  Figure 8 demonstrates the added value of the IoT industry and high- and new-tech industries.

It is obvious that the added value of the high- and new-tech industry is constantly increasing with the development of the IoT industry. In addition, the growth is most prominent in the manufacturing of electronic computers and office equipment. The industrial added value of the electronic computer and office equipment manufacturing industry increased from 31.4 trillion yuan to 56.9 trillion yuan between 2016 and 2021. This shows that the development of the IoT industry has accelerated the development of the high- and new-tech industry.

### 3.2. Analysis of the Impact of the IoT Industry on the Optimization of the High- And New-Tech Industry Structure

Figure 9 shows the gray correlation between the development of the IoT industry and the high- and new-tech industry between 2016 and 2021.

The gray correlation between the development of the IoT industry and the high- and new-tech industry is both 0.64, which shows a strong correlation. From 2016 to 2018, the IoT industry had the strongest correlation with medical equipment and instrument manufacturing, electronic computer and office equipment manufacturing, and electronics and communication manufacturing, with an average of 0.75. From 2018 to 2021, the gray correlation degree of the high- and new-tech industry is decreased. This is related to the development of IoT technology and changes in the structure of the high- and new-tech industry. To sum up, the development of the IoT industry has a strong correlation with the high- and new-tech industry. It exposes that the IoT industry has driven the development of the high- and new-tech industry, thus causing changes in the industrial structure. The optimization analysis of the development of the IoT industry on the structure of the high- and new-tech industry is shown in Figure 10.

With the development of the IoT industry, the output of industrial structure optimization of electronic computer and office equipment manufacturing and electronics and communication manufacturing has a large proportion. The average output ratio of computer and office equipment manufacturing is 47.09%. The average output ratio of the industrial structure optimization of the electronics and communication manufacturing industry is 42.55%. However, the proportion of the output of the industrial structure optimization of medical manufacturing and medical equipment and instrument manufacturing is small, 15.63% and 10.54%, respectively. This shows that the expansion of the IoT industry under the wireless mobile network has been discovered to have a significant impact on the structure optimization of the electronic industry, as well as the structure optimization of the high- and new-tech industries.

## 4. Conclusion

Recent advances in IoT have attracted the attention of researchers and developers all over the world. IoT developers and researchers are collaborating to expand the technology and benefit society to the greatest possible extent. In this study, the changes in the structure of the high- and new-tech industry were investigated by analyzing the changes in the development of the IoT industry under the wireless mobile network. The influence of optimizing the high- and new-tech industry structure was explored using the gray correlation degree to analyze the high- and new-tech industries under the development of the IoT industry. The results showed that the electronics and communication manufacturing industry accounts for the highest proportion of the total output value of the high- and new-tech industry. The electronic computer and office equipment manufacturing industry ranked second. The total output value of the medical manufacturing industry accounted for 13.30%, and the total output value of medical equipment and instrument manufacturing reported was 5.33%. The aerospace equipment manufacturing industry accounted for the lowest share at 2.42%. Similarly, the gray correlation between the development of the IoT industry and the high- and new-tech industry is both 0.64, which showed a strong correlation. This confirmed that with the development of the IoT industry, the industrial structure optimization of high- and new-tech electronic computer and office equipment manufacturing and electronics and communication manufacturing has a larger proportion of output, although this study analyzed the influence of the development of the IoT industry under the wireless mobile network on the optimization of the industrial structure of the high- and new-tech industry in China. However, the development of the IoT industry and the structure of high- and new-tech industries are constantly changing. Researchers can conduct research according to local conditions and the environment. The impact of the IoT sector on the optimization of the high-tech industry structure will be obvious in different places and at different times. [30].

## Figures and Tables

**Figure 1:** Structure of wireless mobile network.

**Figure 2:** Radio resource management.

**Figure 3:** Three layers of the IoT.

**Figure 4:** Theoretical basis for the development of the IoT industry.

**Figure 5:** Contents of industrial structure optimization.

**Figure 6:** Role of the development of the IoT industry in optimizing the structure of high- and new-tech industries.

**Figure 7:** Total output value structure of high-tech industries.

**Figure 8:** Added value of IoT industry and high-tech industry (100 million yuan).

**Figure 9:** Gray correlation between the development of the IoT industry and the high- and new-tech industry.

**Figure 10:** Analysis of the optimization of the high- and new-tech industry structure by the development of the IoT industry.

**Table 1:** Mechanism of industrial structure optimization.

Mechanism	Content
Adjustment of industrial structure (basic)	Adjustment of supply structure and demand structure
Optimization of industrial structure (purpose)	Sophistication and rationalization of industrial structure
Industrial structure effect (influence)	The impact of industrial structure changes on economic growth
National economy (embodiment)	Rapid growth achieved under the positive effect of industrial structure

## Data Availability

The datasets used and/or analyzed during this study are available from the corresponding author upon reasonable request.
